The article "A Precise Medical Imaging Approach for Brain MRI Image Classification" was retracted in 2023. Reasons: signs of a paper mill; compromised peer review; unreliable results or conclusions.

# A Precise Medical Imaging Approach for Brain MRI Image Classification

**DOI:** 10.1155/2022/6447769

**Published:** 2022-05-02

**Authors:** Muhammad Hameed Siddiqi, Ahmed Alsayat, Yousef Alhwaiti, Mohammad Azad, Madallah Alruwaili, Saad Alanazi, M. M. Kamruzzaman, Asfandyar Khan

**Affiliations:** ^1^College of Computer and Information Sciences, Jouf University, Sakaka, Aljouf, Saudi Arabia; ^2^Institute of Computer Science & IT, The University of Agriculture Peshawar, Peshawar, Pakistan

## Abstract

Magnetic resonance imaging (MRI) is an accurate and noninvasive method employed for the diagnosis of various kinds of diseases in medical imaging. Most of the existing systems showed significant performances on small MRI datasets, while their performances decrease against large MRI datasets. Hence, the goal was to design an efficient and robust classification system that sustains a high recognition rate against large MRI dataset. Accordingly, in this study, we have proposed the usage of a novel feature extraction technique that has the ability to extract and select the prominent feature from MRI image. The proposed algorithm selects the best features from the MRI images of various diseases. Further, this approach discriminates various classes based on recursive values such as partial *Z*-value. The proposed approach only extracts a minor feature set through, respectively, forward and backward recursion models. The most interrelated features are nominated in the forward regression model that depends on the values of partial *Z*-test, while the minimum interrelated features are diminished from the corresponding feature space under the presence of the backward model. In both cases, the values of *Z*-test are estimated through the defined labels of the diseases. The proposed model is efficiently looking the localized features, which is one of the benefits of this method. After extracting and selecting the best features, the model is trained by utilizing support vector machine (SVM) to provide the predicted labels to the corresponding MRI images. To show the significance of the proposed model, we utilized a publicly available standard dataset such as Harvard Medical School and Open Access Series of Imaging Studies (OASIS), which contains 24 various brain diseases including normal. The proposed approach achieved the best classification accuracy against existing state-of-the-art systems.

## 1. Introduction

As per the new report of United Nations, nearly one in every six people or up to 1 billion people on the planet suffer from neurological disorders such as Alzheimer's and Parkinson's diseases, strokes, multiple sclerosis, and epilepsy, as well as migraine, brain injuries, and neuro-infections, with 6.8 million people dying each year [1].

The article "A Precise Medical Imaging Approach for Brain MRI Image Classification" was retracted in 2023. Reasons: signs of a paper mill; compromised peer review; unreliable results or conclusions.

Medical imaging is the procedure of utilizing the technology to assess the humans in the awareness of analyzing, monitoring, and treating medical concerns. Some of the well-known medical approaches such as magnetic resonance imaging (MRI), positron emission tomography (PET), and computed tomography (CT) are commonly utilized in healthcare systems. However, MRI is one of the best candidates utilized for brain diseases. Among this imaging, MRI is an accurate and noninvasive method employed for the diagnosis of various kinds of diseases in medical imaging. Mostly, MRI is beneficial for the processing of soft tissues. Hence, MRI permits the significant brain imaging with the best anatomic aspect and suggests more sensitivity and specificity than other imaging systems for various kinds of neurologic situations.

The radiologists' conservative procedure for the classification of brain MRI images is visual examination [2]. However, due to the large scale of imagery data, the previous heuristic calculations of investigation and understanding of such compositions are monotonous, time overwhelming, expensive, and do not encapsulate the entire outline of shrivel. Therefore, it produces the necessity of proposing automatic identification frameworks for the investigation and recognition of brain MRI images. These systems might be an excessive tool for the medical diagnosis and premedical and post-medical processes [3–7].

In the literature, many scholars have designed different kinds of techniques for brain MRI classification. Most of these approaches consist of three modules such as feature extraction, feature selection, and classification in a brain MRI classification system. The authors of [8] utilized an inception residual network on a publicly brain MRI dataset and achieved 69% classification accuracy. In [9], the authors utilized deep learning coupled with data hungry network to classify the brain MRI image. They achieved 42% accuracy of classification. Similarly, a recent system was proposed by [10] for the classification of brain disease, which was based on relevance-guided deep learning. Likewise, in [11], the authors segmented the tumor from brain MRI images, which was based on a lightweight deep model. They achieved 91% against the brain MRI image dataset. A recent work was proposed by [12] that was based on AlexNet and GoogleNet, which were trained on a huge amount of real dataset, and claimed 89% of classification. On the other hand, a state-of-the-art work was proposed by [13], where they extracted the shape-based and texture-based features by utilizing the wavelet transform and histogram of oriented gradient, respectively. For classification purpose, they employed one of the well-known machine learning algorithms such as random forest. Moreover, in their work, they extracted the abnormal brain tissues in low contrast. They claimed the highest accuracy against the real dataset. The authors of [14] classified the brain MRI images by utilizing three various classification methods such as pretrained Inception V3, ResNet50, and VGG-16. The entire images were preprocessed to improve the efficiency of their system. They attained 94% recognition rate against the MRI dataset. Furthermore, a novel framework was designed by [15] for the brain tumor detection against various MRI datasets. This framework was based on transfer learning methods and fully convolutional neural network model, which has five steps such as pre- and post-processing, skull denudation, segmentation, and classification. They achieved the highest accuracy of classification. However, most of these systems showed significant performances and achieved higher recognition rates on small MRI datasets, but their performances decrease against large MRI datasets. Hence, the goal is to design an efficient and robust classification system that sustains high recognition rate against large MRI dataset.

The article "A Precise Medical Imaging Approach for Brain MRI Image Classification" was retracted in 2023. Reasons: signs of a paper mill; compromised peer review; unreliable results or conclusions.

Accordingly, in this research, we have proposed the usage of a new feature extraction algorithm named stepwise linear discriminant analysis. This algorithm has the ability to extract and select the prominent features from the MRI images of various diseases. This method focuses on the selection of the best features from MRI images and discriminating the corresponding classes (different diseases) through the value of regression such as *Z*-value. The proposed approach only extracts a minor feature set through, respectively, forward and backward recursion models. The most interrelated features are nominated in the forward regression model that depends on the values of partial *Z*-test, while the minimum interrelated features are diminished from the corresponding feature space under the presence of backward model. In both cases, the values of *Z*-test are estimated through the defined labels of the diseases. The proposed model is efficiently looking the localized features, which is one of the benefits of this method. After extracting and selecting the best features, the model is trained by utilizing support vector machine (SVM) to provide the predicted labels to the corresponding MRI images. The significance of the developed technique is justified against a benchmark MRI dataset. A generalized dataset is gathered from Harvard Medical School [16] and Open Access Series of Imaging Studies (OASIS) [17]. This dataset consists of 24 brain diseases including normal brain (NB). The diseases are glioma (GL), sarcoma (SR), fatal stroke (FT), multiple embolic infarctions (MIs), motor neuron (MN) sickness, multiple sclerosis (MS), vascular dementia (VD), cavernous angioma (CA), cerebral calcinosis (CC), chronic subdural (CS) hematoma, cerebral haemorrhage (CH), Alzheimer's (AL) sickness, Huntington's disease (HD), AIDS dementia (AD), Pick's disease (PD), metastatic adenocarcinoma (MA), hypertensive encephalopathy (HY), Alzheimer's sickness with visible agnosia (AV), Creutzfeldt–Jakob (CJ) sickness, cerebral toxoplasmosis (CT), Lyme encephalopathy (LE), herpes encephalitis (HE), meningioma (M), and metastatic bronchogenic (MB) carcinoma. The proposed approach achieved the best classification accuracy against existing state-of-the art systems.

The article "A Precise Medical Imaging Approach for Brain MRI Image Classification" was retracted in 2023. Reasons: signs of a paper mill; compromised peer review; unreliable results or conclusions.

The remaining study is arranged as follows: Section 2 shows the latest existing systems with their shortcomings against the MRI image dataset. In Section 3, we have provided a comprehensive description of the proposed technique followed by support vector machine, while in Section 4, the experimental setup is presented. The corresponding results are indicated in Section 5. Finally, in Section 6, we summarize the study with some future directions.

## 2. Related Work

In the literature, many scholars have designed different kinds of techniques for brain MRI classification. However, most of these systems showed significant performances and achieved higher recognition rates on small MRI datasets, but their performances decrease against large MRI datasets. Hence, the goal was to design an efficient and robust classification system that sustains a high recognition rate against large MRI dataset.

A state-of-the art algorithm was proposed by [18], where the authors clustered the brain MRI images to detect and locate the brain tumor. For clustering, they utilized an unsupervised principal component analysis (PCA) to achieve the best results. However, the major limitation of the PCA is that it is a least-squares method that flops to account for outliers [19]. Moreover, they utilized only five brain diseases, and for each disease, only ten images are considered. Similarly, a new algorithm was developed by [20] for the classification of various brain diseases against MRI images. They employed wavelet transform for feature extraction, while for classification, they utilized a support vector machine. In their systems, they considered only seven common brain diseases. However, wavelet transform is categorized through lack of alignment discrimination and shift modification. Moreover, the coefficients of the wavelet transform suffer from the aliasing effect [21].

The article "A Precise Medical Imaging Approach for Brain MRI Image Classification" was retracted in 2023. Reasons: signs of a paper mill; compromised peer review; unreliable results or conclusions.

On the other hand, a multilevel support vector machine-based system was developed by [22] for brain tumor detection. There are four modules in this system: image acquisition, preprocessing, feature extraction, and classification. The classification rate for the system was 85% between normal and abnormal. However, this system presumes that the data are identical and independently distributed, which is obviously not in image voxels. Mostly, the labels of the voxels are strongly relied on their surrounding points [23]. Likewise, a novel method was designed by [24] based on a deep wavelet autoencoder to resolve the performance, validation, and long-term processing issues against brain MRI images. However, the deep wavelet autoencoder has poor directionality, is complex to variations, and lacks phase information, and the resultant MRI slices might not attain the foci of the disease [25]. A robust architecture was developed by [26] for segmentation against brain MRI, which was based on patch-wise U-Net. In this architecture, the MRI slices are divided into non-overlying patches, which are nourished inside the model coupled with their appropriate patches of the data so in respect of training the network. However, the U-Net model has weak generalization capability, which means that it does not have the ability to learn the deep information [27]. To solve the limitation of U-Net, the authors of [28] developed an M-Net architecture for brain MRI segmentation. This model consists of left and right, encoding and decoding tracks, which help the model extract the best features from the brain MRI images. However, M-Net has common drawbacks while taking a comprehensive image as an input [27].

A state-of-the art convolutional dictionary learning with the local constraint method was proposed by [29] for the classification of brain tumor against the MRI dataset. In this system, the discriminatory data were discovered through multilayer dictionary learning. A trained kNN-based graph was utilized to preserve the symmetrical structure of the data, due to which the difference in the attained dictionary is solid. However, for each variable, kNN requires suitable values from corresponding data [30]. A recent multi-convolutional neural network-based system was developed by [31] for the early diagnosis of brain tumor. In this system, they employed three convolutional neural network (CNN) models for three various types of tasks, where the individual model was utilized for brain tumor detection, classification of tumor disease, and classification of tumor grades, respectively. A hybrid approach was developed by [32] to classify normal and abnormal MRI images.

The article "A Precise Medical Imaging Approach for Brain MRI Image Classification" was retracted in 2023. Reasons: signs of a paper mill; compromised peer review; unreliable results or conclusions.

The approach utilized well-known existing methods such as wavelet transform, principal component analysis (PCA), and back propagation. Wavelet transform was used to extract the best features, while PCA was utilized to reduce the dimension of the feature space and to find the optimum weight of the mode, and back propagation was employed in the model. However, wavelet transform is categorized through lack of alignment discrimination and shift modification. Moreover, the coefficients of the wavelet transform suffer from the aliasing effect [21]. Moreover, one of the major limitations of PCA is that it is a least-squares method that flops to account for outliers [19]. Also, the back propagation has a common limitation, which does not guarantee to find the global minimum of the error function.

An effective mechanism was designed by [33] for the brain MRI segmentation. In this mechanism, a self-learning network was utilized for the real brain MRI images. However, they utilized a small dataset for the experiments, and the system did not show significant performance as well. An integrated system was developed by [34], which was based on the Haar wavelet transform and convolutional neural network. They utilized a median filter for enhancement and multilevel Haar wavelet transform for feature extraction. Moreover, in this step, they diminished the unnecessary details and reduced the size of the MRI images. In the final step, they employed a convolutional neural network to classify normal and abnormal MRI. However, the main limitation of the Haar wavelet transform is feature cutoff, which leads to problems in simulating continuous signals [35]. Another integrated approach was developed by [36], where the authors employed wavelet transform, PCA, and artificial neural network for the purpose of MR classification. However, PCA and wavelet transform have their own limitations, which are described in [19, 21], respectively. Another latest framework was proposed by [37] against MRI images, which was based on the convolution neural network. The framework was utilized in health care for the brain tumor diagnosis.

A novel integrated clustering approach was developed by [38], where the authors employed *K*-mean coupled with spatial fuzzy C-mean clustering algorithms. Moreover, they also utilized wavelet transform for feature extraction. The constant size is required for centroids that collect the data using K-mean during the process, and the generation of the cluster is empty [39]. Similarly, the authors of [40] developed a multinomial logistic regression-based approach for the classification of Alzheimer's diseases. They provided a general classification framework for mild Alzheimer's disease, moderate, non-demented, and very mild. However, logistic regression might not be used if the number of observations is smaller than the number of the corresponding features; otherwise, it might produce overfitting.

The article "A Precise Medical Imaging Approach for Brain MRI Image Classification" was retracted in 2023. Reasons: signs of a paper mill; compromised peer review; unreliable results or conclusions.

Accordingly, in this study, we have designed an accurate and efficient approach for brain MRI classification system that has the ability to extract and select the best features from the brain MRI images. The proposed method extracts and selects the prominent features by considering the benefit forward selection technique. Moreover, the proposed method also takes the benefit of backward regression technique to diminish the unwanted features from the brain MRI images.

## 3. Proposed Edge Detection Algorithm

Figure 1 depicts the overall strategy.

### 3.1. Stepwise Linear Discriminant Analysis

We will talk about the Fisher linear discriminant (FLD) in this part, which is a well-known linear classification method for separating two classes [41]. For two classes with the same covariance, the Gaussian distribution approach can be employed; however, FLD is a more robust classifier for determining the optimal separation between the classes. FLD is a method that is comparable to regression methods such as least-squares regression, and it projects feature masses in binary jobs as follows:

(1) $$\begin{array}{c} \tilde{C}=\;{\left(P^{t}P\right)}^{-1}P^{t}y, \end{array}$$

where $\tilde{C}$ is the label of the class and *P* is the pragmatic feature vector matrix. FLD's ability to produce good classification results is limited to linear data. We developed a stepwise linear discriminant analysis (SWLDA) as a way to cope with nonlinear classification techniques, which was validated using the P300 Speller response [42]. In comparison with FLD, SWLDA works in parallel, decreasing feature space and deleting unnecessary features.

SWLDA was used to choose the best features utilizing two algorithms, forward and backward algorithms that worked in parallel. The model “*Z*-value 0.15” was the most significant value found when there was no initial model. The incorrect values were deleted using the backward algorithm (such as “*p* values >0.2”) after the values were entered using the forward algorithm. This process is repeated until the predefined condition is met, and the resulting function is limited to 100 attributes.

The forward regression approach selects the best variables, such as *X*, and then moves on to significantly increase the number of *X*s. The process of adding new entries and selecting values is influenced by the *Z*-test value, which determines which entry should be inserted first. Following that, a comparison is performed between two values: partial *Z*-value and selected value. Throughout the process, the forward technique is used. Backward regression is used to do the deletion procedure (known as backward deletion). The testing (*Z*-test) that was in the backlog is calculated during this phase. In the case of the testing value being the lowest one, then *V*_*L*_ is differentiated with the preselected value, *P*_*S*_. Then:

- If *V*_*L*_ < *P*_*S*_, the *Z*-test calculation will begin again.
- Otherwise, the regression equation is accepted.

The article "A Precise Medical Imaging Approach for Brain MRI Image Classification" was retracted in 2023. Reasons: signs of a paper mill; compromised peer review; unreliable results or conclusions.

The model is developed to demonstrate iterations using stepwise regression. There are automatic selections of independent variables in each iteration. SWLDA based on stepwise regression incorporates all independent variables and excludes those that are not statistically significant from the stepwise model [40]. The working for forward selection and backward removal models with five variables are presented in Figures 2 and 3.

### 3.2. Implementation of SWLDA

At the beginning of the SWLDA model, there are no predictor variables. In each step, predictor variables are either included or excluded from the model based on the significance test, i.e., partial *F*-tests (the *t*-tests). For the significance level test, two variables are defined: alpha-to-included and alpha-to-excluded. The threshold parameters are alpha-to-included *α*_*i*_ = 0.15 and alpha-to-excluded *α*_*e*_ = 0.2. The importance of the predictor variable that is included or excluded from the model is also displayed at this level. When there are no more predictors that can be included or excluded from the stepwise model, the algorithm stops iterating.

For example, “*p*” denotes the number of input variables *x*_1_, *x*_2_, *x*_3_,…, *x*_*p*_. Let “*y*” be the output variable. Regression is a technique for fitting variables into a model, such as regress *y* on *x*_1_, regress *y* on *x*_2_ … and regress *y* on *x*_*p−*1_. The stepwise model starts with the predictor with the smallest *t*-test *p* value, i.e., below *α*_*i*_ = 0.15. This procedure is repeated until the stopping criteria are met; i.e., there are no variables with a *p* value smaller than *α*_*i*_. Let *x*_*1*_ be the most accurate predictor.

Next, we fit the remaining predictor model to the best predictor *x*_1_ in the model, i.e., regress *y* on (*x*_1_, *x*_2_), regress *y* on (*x*_1_, *x*_3_) … regress *y* on (*x*_1_, *x*_*p*−1_). The predictor with the lowest *p* value (*α*_*i*_ = 0.15) is inserted into the stepwise model in the second stage. When there is no *p* value smaller than 0.15, the loop ends once more. Let *x*_*2*_ be the “best second predictor” in the model. The program takes a step back and examines the *p* value for *γ*_1_ = 0, that is, the predictor variable removal criteria from the model. If the p value has (above *α*e = 0.2) for *γ*1 = 0, then the variable is regarded as not significant when compared to the new entry. Consider the case where both variables *x*_1_ and *x*_2_ are included in the two-predictor stepwise model. The method then fits each of the three-predictor models with *x*_1_ and *x*_2_ in the model, i.e., regress *y* on (*x*_1_, *x*_2_, *x*_3_) and regress *y* on (*x*_1_, *x*_2_, *x*_4_),…, and regress *y* on (*x*_1_, *x*_2_, *x*_*p*−1_). The predictor with the least *p* value (<*α*_*i*_ = 0.15) is the third predictor to enter the stepwise model. When there is no *p* value <*α*_*i,*_ the stopping requirement is met. The algorithm checks the *p* values for *γ*_1_ = 0 in this scenario. Predictor is eliminated from the stepwise model if either of the *p* values has become nonsignificant (above *α*_*e*_ = 0.2). When adding a new predictor does not result in a *p* value less than *α*_*i*_ = 0.15, the algorithm ends.

The article "A Precise Medical Imaging Approach for Brain MRI Image Classification" was retracted in 2023. Reasons: signs of a paper mill; compromised peer review; unreliable results or conclusions.

In short, the proposed approach is a method of choosing appropriate predictor variables to include a multiple regression model. The linear discriminant and least-squares regression solutions are identical for binary classification tasks like this. Stepwise regression is used in both forward and backward directions. The most statistically significant predictor variable with a *p* value less than 0.1 is added to the model after it has no initial model terms. A backward stepwise regression is done after each new addition to the model to remove the least significant variables with *p* values >0.15. This procedure is repeated until the model containing a preset number of terms or no more terms meets the inclusion/exclusion criteria.

### 3.3. Classification via Support Vector Machine

One of the most well-known numerical approaches for image processing, pattern recognition, and machine intelligence is the support vector machine (SVM) [44]. SVM is widely utilized in the classification of linear and twofold data. It is based on the best splitting option hyperplane between two or more classes, as well as the supreme boundary inside each class' shapes. SVM uses the ostensible goal of projecting data from a single feature space to a higher-dimensional space, resulting in linear classification in the novel space equaling nonlinear classification in the original space.

Using hyperplanes, SVM may identify two or more classes. We used an optimal technique to find the best separating hyperplane within distinct class symbols in this step, as shown in Figure 4. SVM is commonly described as follows:

(2) $$\begin{array}{c} \left(\overset{⟶}{R},\;µ\left(t\right)\right)+\;D\;=\;0, \end{array}$$

where $\overset{⟶}{\text{R}}$ is the usual vector to the hyperplane that partitions the two or more classes, *µ* is the function of the inserting data, *t* is the data point, and *D* is the training data. As shown below, this is linked to the next function:

(3) $$\begin{array}{c} \overset{⟶}{S}\left(t\right)=\;signi\left(\left(R,\;µ\left(t\right)\right)+\;D\right). \end{array}$$

where $\overset{⟶}{\text{S}}\left(\text{t}\right)$ is the next function that displays the training designs; this is the so-called support vector that holds all of the data in the vicinity of the classification concerns. See SVM [44] for further information.

The article "A Precise Medical Imaging Approach for Brain MRI Image Classification" was retracted in 2023. Reasons: signs of a paper mill; compromised peer review; unreliable results or conclusions.

## 4. Designed Approach Evaluation

The proposed technique is evaluated in the following order to show the performance of the proposed technique.

### 4.1. MRI Dataset

For this research, we have gathered a generalized MRI dataset from, respectively, Harvard Medical School and OASIS MRI datasets, which contains original MRI images from 340 real patients (male and female). The dataset has, respectively, T1- and T2-weighted brain MRI images. The entire patients are right-handed, and the size of every image size is 256 × 256 with demographic and clinical details such as gender, age, clinical dementia rating, observation of mental state, and parameters of various tests. This dataset is divided into two groups, the first group contains eleven diseases (which is utilized by most of the existing works as a benchmark dataset), while the other group consists of 24 diseases including eleven from the group 1. This group is more universal for comprehensive experiments. There are a total of 255 brain MRI images in the first group (220 abnormal and 35 normal images), while the second group has total 340 images (260 abnormal and 80 normal images, respectively). The sample images for these diseases are shown in Figure 5.

### 4.2. Experimental Arrangement

The proposed algorithm is evaluated against the following series of experiments. All the experiments are executed in MATLAB with the specification of 8 GB RAM and 1.7 Hz.

- The first experiment represents the accuracy of the proposed algorithm against the MRI dataset.
- In the second experiment, we performed a series of sub-experiments to show the effectiveness of the proposed technique. For these sub-experiments, we utilized existing well-known methods such as independent component analysis, Isomap, kernel principal component analysis, latent semantic analysis, partial least squares, multifactor dimensionality reduction, nonlinear dimensionality reduction, multilinear principal component analysis, multilinear subspace learning, and semidefinite embedding instead of using the proposed technique.
- In the third sub-experiment, the recognition rate of the proposed technique is compared against state-of-the-art systems.

The article "A Precise Medical Imaging Approach for Brain MRI Image Classification" was retracted in 2023. Reasons: signs of a paper mill; compromised peer review; unreliable results or conclusions.

## 5. Designed Approach Evaluation

The entire experiments are described in the following order to show the performance of the proposed approach.

### 5.1. 1st Experiment

In this experiment, the effectiveness of the proposed algorithm is assessed against the MRI dataset. For this experiment, we employed *n*-fold cross-validation scheme, which means that every image is used for training and testing, respectively. The overall results are represented in Table 1.

It is clear from Table 1 that the proposed algorithm achieved significant accuracy of classification against the MRI dataset. This is because the suggested algorithm is efficient and selects acceptable features in a non-exhaustive way, resulting in the heuristic implementation being terminated. The only required parameters, the maximum model order and termination heuristic, are intuitive and can be easily estimated based on the expected data properties. In several ways, the proposed technique benefits from automatic feature extraction. Because irrelevant terms are deleted from the model (i.e., weights are set to zero), utilizing less training data reduces the likelihood of the classification result being tainted.

### 5.2. 2nd Experiment

In the second experiment, we have performed a comprehensive set of sub-experiments to show the importance of the proposed algorithm. For these sub-experiments, we utilized existing well-known feature extraction and selection methods instead of employing the proposed technique. These methods are accordingly implemented based on their respective settings. Some methods have been implemented, while for some methods, we have borrowed their implementations, and for the remaining methods, we have used their results as presented in their articles. The overall results are represented in Tables 2–11.

It is clearly described in Tables 2–11 that without using the proposed algorithm, the system did not achieve the best accuracy of classification. From these sub-experiments, we can judge the significance of the proposed algorithm in the classification of various types of diseases against MRI images. This is because the proposed approach has the ability to extract and select the best features from the brain MRI images. The proposed method extracts and selects the prominent features by considering the benefit forward selection technique. Moreover, the proposed method also takes the benefit of backward regression technique to diminish the unwanted features from the brain MRI images.

The article "A Precise Medical Imaging Approach for Brain MRI Image Classification" was retracted in 2023. Reasons: signs of a paper mill; compromised peer review; unreliable results or conclusions.

### 5.3. 3rd Experiment

In this experiment, the accuracy of the proposed technique is compared with the latest existing methods against MRI images. These methods are accordingly implemented based on their respective settings. Some methods have been implemented, while for some methods, we have borrowed their implementations, and for the remaining methods, we have used their results as presented in their articles. The overall results are described in Table 12.

It can be assessed from Table 12 that the proposed approach showed the best accuracy against state-of-the-art methods on a publicly available standard MRI dataset. This is because the proposed approach considers the benefits of the forward and backward models. Accordingly, this algorithm selects the best features from the MRI images of various diseases. Further, this approach discriminates various classes based on recursive values such as partial *Z*-value. The proposed approach only extracts a minor feature set through, respectively, forward and backward recursion models. The most interrelated features are nominated in the forward regression model that depends on the values of partial *Z*-test, while the minimum interrelated features are diminished from the corresponding feature space under the presence of backward model. In both cases, the values of *Z*-test are estimated through the defined labels of the diseases. The proposed model is efficiently looking the localized features, which is one of the benefits of this method.

## 6. Conclusion

Magnetic resonance imaging is an imperative diagnostic method for the initial detection and classification of various brain diseases from MRI images, which is one of the challenging tasks because of various shapes, positions, and intensities of brain cells. Many researchers have developed various strategies for brain MRI categorization. On short MRI datasets, however, the majority of these systems performed well and had greater recognition rates. However, when it comes to large MRI datasets, their performance suffers. As a result, the goal is to create a fast and reliable classification system that can maintain a high recognition rate across a huge MRI dataset. We propose in this work the use of a unique feature extraction technique that can extract and pick the most prominent feature from an MRI image. The suggested algorithm picks out the most important elements from MRI pictures of various disorders. Furthermore, this method distinguishes between multiple classes based on recursive values such as partial Z-value. Through forward and backward recursion models, the suggested method only extracts a tiny feature set. In a forward regression model based on partial *Z*-test values, the most interrelated features are nominated, whereas in a backward regression model, the least interrelated features are reduced from the corresponding feature space. The values of the *Z*-test are estimated in both situations using the diseases' stated labels. One of the advantages of this strategy is that it searches for localized features quickly. The model is trained using support vector machine (SVM) to offer predicted labels to the relevant MRI images after extracting and selecting the best attributes. We used a publicly available standard dataset from Harvard Medical School and Open Access Series of Imaging Studies (OASIS), which covers 24 different brain illnesses, including normal, to demonstrate the significance of the suggested approach. In comparison with the existing state-of-the-art systems, the proposed technique attained the highest classification accuracy.

The article "A Precise Medical Imaging Approach for Brain MRI Image Classification" was retracted in 2023. Reasons: signs of a paper mill; compromised peer review; unreliable results or conclusions.

The majority of existing MRI image classification methods were developed in a laboratory setting, which is not practical. As a result, in the future, we are planning to use the proposed system, as well as the proposed feature extraction approach, in health care to help medical specialists and physicians.

## Figures and Tables

**Figure 1:** Flowchart of the proposed MRI image classification system.

**Figure 2:** Example of forward stepwise selection with five variables [43].

**Figure 3:** Example of backward stepwise deletion with five variables [43].

**Figure 4:** Optimal scattering hyperplane [44].

**Figure 5:** Sample images from the generalized brain MRI dataset, where every image represents the individual brain disease [2].

**Table 1:** Classification results of the proposed algorithm against the brain MRI dataset (unit %).

Diseases	NB	GL	SR	AL	AV	PD	HD	M	CS	MS	CT	HE	MB	MA	MN	CC	AD	LE	CJ	HY	MI	CH	CA	VD	FT
NB	**96**	0	0	1	0	0	0	1	0	0	0	0	0	0	0	0	0	1	0	0	0	0	0	1	0
GL	1	**95**	0	0	0	1	0	0	0	0	0	2	0	0	0	0	0	0	0	1	0	0	0	0	0
SR	0	1	**97**	0	0	0	0	0	0	0	0	0	0	0	1	0	0	0	0	0	0	0	0	0	1
AL	0	0	0	**99**	0	0	0	0	1	0	0	0	0	0	0	0	0	0	0	0	0	0	0	0	0
AV	0	0	0	0	**100**	0	0	0	0	0	0	0	0	0	0	0	0	0	0	0	0	0	0	0	0
PD	0	2	0	0	0	**94**	0	0	0	0	0	1	0	0	0	0	0	1	0	0	0	0	0	2	0
HD	1	0	0	0	2	0	**92**	0	1	0	0	0	0	0	1	0	0	0	2	0	0	1	0	0	0
M	0	0	1	0	0	0	0	**96**	0	0	0	0	1	0	0	0	1	0	0	0	0	0	1	0	0
CS	0	0	0	0	0	0	1	0	**98**	0	0	0	0	0	0	0	0	0	0	1	0	0	0	0	0
MS	1	0	0	0	0	0	0	0	0	**99**	0	0	0	0	0	0	0	0	0	0	0	0	0	0	0
CT	0	0	0	0	0	0	0	0	0	0	**100**	0	0	0	0	0	0	0	0	0	0	0	0	0	0
HE	0	0	2	0	0	0	0	0	1	0	0	**94**	0	0	0	1	0	0	0	0	0	0	0	0	2
MB	1	0	0	0	0	2	0	0	0	0	1	0	**92**	1	0	0	0	0	1	0	0	0	2	0	0
MA	0	1	0	0	0	0	0	2	0	0	0	0	0	**95**	0	0	0	1	0	0	1	0	0	0	0
MN	0	0	0	1	0	0	0	0	0	1	0	0	0	0	**96**	0	0	0	0	1	0	0	0	1	0
CC	1	0	0	0	0	0	0	0	0	0	0	0	0	0	2	**97**	0	0	0	0	0	0	0	0	0
AD	0	0	1	0	0	0	0	0	0	0	0	0	0	0	0	0	**99**	0	0	0	0	0	0	0	0
LE	0	0	0	0	0	1	0	0	0	0	0	0	1	0	0	0	0	**98**	0	0	0	0	0	0	0
CJ	1	0	0	0	0	0	0	0	2	0	0	0	0	0	0	0	1	0	**96**	0	0	0	0	0	0
HY	0	2	0	0	0	0	1	0	0	0	0	0	0	1	0	0	0	0	0	**94**	0	0	1	0	1
MI	0	0	0	2	0	0	0	0	0	1	0	0	0	0	0	1	0	0	1	0	**93**	0	0	2	0
CH	0	0	0	0	0	0	0	0	0	0	0	1	0	0	0	0	0	0	0	0	0	**99**	0	0	0
CA	1	0	0	0	1	0	0	0	0	0	0	0	0	0	1	0	0	0	0	0	1	0	**96**	0	0
VD	0	0	1	0	0	0	0	1	0	0	0	0	0	0	0	0	0	2	0	0	0	1	0	**95**	0
FT	0	0	0	0	0	0	0	0	0	0	0	0	0	0	0	0	0	0	0	0	0	0	0	0	**100**

Average	96.40%																								

The bold values are to differentiate the original results from the missing results.

The article "A Precise Medical Imaging Approach for Brain MRI Image Classification" was retracted in 2023. Reasons: signs of a paper mill; compromised peer review; unreliable results or conclusions.

**Table 2:** Classification results of independent component analysis (without using the proposed technique) on the brain MRI dataset (unit %).

Diseases	NB	GL	SR	AL	AV	PD	HD	M	CS	MS	CT	HE	MB	MA	MN	CC	AD	LE	CJ	HY	MI	CH	CA	VD	FT
NB	**78**	0	2	0	1	1	0	2	0	4	0	1	0	2	0	0	1	0	0	0	4	0	0	2	2
GL	4	**70**	0	2	0	2	2	0	1	0	1	0	2	0	6	1	0	2	0	2	0	1	0	0	4
SR	0	2	**71**	0	4	0	1	1	0	6	0	2	0	4	1	0	2	0	2	0	2	0	1	1	0
AL	2	0	0	**75**	2	1	0	0	4	0	1	0	2	0	1	1	0	4	0	1	0	1	4	0	1
AV	0	1	4	0	**73**	0	2	2	0	2	1	1	0	2	0	0	4	0	2	0	1	0	0	1	4
PD	6	0	1	2	0	**70**	0	0	2	0	2	0	4	0	2	2	0	2	1	2	0	1	1	1	1
HD	2	2	0	0	4	0	**72**	4	0	1	0	2	0	1	1	0	1	0	6	0	2	0	0	2	0
M	0	2	2	1	0	2	0	**77**	2	0	4	0	2	0	0	1	0	2	0	1	0	1	1	0	2
CS	1	0	2	0	2	0	1	1	**75**	4	0	2	0	1	2	0	2	0	2	0	2	0	1	1	1
MS	2	2	0	4	0	2	0	1	1	**71**	2	1	1	0	0	6	0	1	0	1	0	2	0	3	0
CT	0	1	2	0	2	0	1	0	2	1	**80**	0	0	2	1	0	2	0	2	0	2	0	1	0	1
HE	1	0	0	2	0	1	0	2	0	0	2	**81**	1	0	0	2	0	1	0	1	0	2	0	2	2
MB	0	2	1	0	2	0	1	0	1	2	0	1	**82**	0	2	0	1	0	1	0	2	0	2	0	0
MA	2	0	0	1	0	2	0	1	0	0	1	2	0	**85**	0	1	0	0	0	2	0	1	0	0	2
MN	0	4	1	0	2	0	1	0	1	1	0	0	2	1	**77**	0	2	2	1	0	1	0	2	2	0
CC	2	0	1	2	0	2	0	2	1	0	2	1	1	0	1	**79**	0	1	0	2	0	0	0	1	2
AD	0	1	0	1	1	0	2	0	0	2	0	0	1	2	0	1	**83**	0	2	0	2	0	1	1	0
LE	1	0	4	0	0	2	0	2	1	0	2	1	0	0	2	0	6	**74**	0	2	0	1	1	0	1
CJ	1	2	0	2	2	0	1	0	0	1	0	0	2	1	0	1	0	0	**82**	0	2	0	0	2	1
HY	2	0	2	0	0	2	0	1	1	0	1	2	0	0	1	0	2	2	0	**81**	0	2	1	1	0
MI	0	1	0	2	1	0	1	0	0	2	0	0	2	0	0	1	0	0	1	1	**84**	0	0	2	2
CH	2	1	2	0	1	2	0	2	1	0	2	1	0	1	2	0	1	1	0	2	1	**76**	1	0	1
CA	1	2	0	2	0	0	2	0	0	2	1	0	2	0	1	2	0	0	2	1	0	2	**78**	2	0
VD	0	1	2	0	2	2	0	1	1	0	0	2	0	1	0	0	2	1	0	0	1	0	1	**83**	0
FT	2	0	0	2	1	0	2	0	0	2	1	0	1	0	2	0	0	2	1	2	0	2	0	1	**79**

Average	77.44%																								

The bold values are to differentiate the original results from the missing results.

**Table 3:** Classification results of Isomap (without using the proposed technique) on the brain MRI dataset (unit %).

Diseases	NB	GL	SR	AL	AV	PD	HD	M	CS	MS	CT	HE	MB	MA	MN	CC	AD	LE	CJ	HY	MI	CH	CA	VD	FT
NB	**65**	2	0	4	2	0	6	1	1	0	2	4	1	0	2	2	0	2	0	1	2	2	1	0	0
GL	2	**70**	1	2	0	2	2	1	0	2	1	0	2	1	0	2	1	0	4	2	0	1	0	2	2
SR	1	4	**69**	0	2	1	0	4	2	1	0	2	0	2	2	0	2	1	1	0	2	1	2	0	1
AL	0	1	2	**73**	1	0	2	0	1	2	4	0	2	0	3	1	0	2	0	2	1	0	1	0	2
AV	2	0	0	1	**74**	2	0	1	2	0	1	2	0	2	2	0	2	1	1	0	1	4	0	2	0
PD	1	2	1	0	2	**75**	1	0	1	2	0	1	1	2	0	2	1	0	2	1	0	1	2	0	2
HD	0	1	0	2	0	2	**77**	2	0	1	1	2	0	1	2	0	1	2	0	1	2	0	0	1	2
M	4	0	2	3	1	0	2	**68**	2	0	2	1	2	0	4	2	0	1	2	0	0	2	1	0	1
CS	1	2	0	1	2	2	0	2	**71**	1	2	0	3	2	0	1	2	0	0	2	2	0	2	2	0
MS	2	1	3	0	1	0	2	0	4	**72**	0	2	0	1	2	0	1	2	0	1	1	2	0	1	2
CT	2	2	0	2	0	4	0	1	1	2	**73**	0	2	0	1	2	0	1	2	1	0	1	2	0	1
HE	0	2	4	0	1	0	2	2	0	1	2	**68**	1	2	0	1	1	0	1	2	2	0	4	2	2
MB	4	0	1	2	0	2	0	1	2	0	2	6	**66**	3	2	0	0	2	1	0	1	2	0	2	1
MA	1	2	0	0	2	0	4	0	1	2	0	1	2	**73**	0	2	1	1	0	2	0	0	2	0	4
MN	2	0	2	4	0	1	1	2	0	0	2	0	1	2	**75**	1	0	2	0	0	2	1	0	2	0
CC	0	2	0	1	2	0	2	1	0	2	1	2	0	1	2	**69**	2	0	4	2	0	0	2	0	5
AD	2	0	1	0	1	2	0	2	4	0	1	1	2	0	2	2	**74**	1	0	0	2	2	0	0	1
LE	0	2	0	2	0	2	4	0	0	2	2	0	0	2	1	0	2	**73**	2	0	2	1	0	1	2
CJ	2	1	4	0	2	0	0	6	2	0	0	4	2	0	2	1	1	0	**67**	2	0	0	4	0	0
HY	0	2	0	1	0	4	2	0	0	6	2	0	0	4	1	0	0	2	1	**69**	2	1	0	2	1
MI	2	0	1	0	2	0	1	2	3	0	0	2	1	0	0	2	4	0	0	2	**72**	0	2	0	4
CH	1	2	0	2	0	2	2	0	1	2	1	0	0	2	2	0	0	1	2	0	1	**75**	2	2	0
CA	2	0	4	0	2	0	0	1	2	0	0	2	1	0	1	3	2	0	4	1	2	0	**71**	0	2
VD	0	1	0	2	0	1	2	0	0	4	2	0	4	2	1	0	0	2	0	2	0	6	2	**68**	1
FT	2	0	1	0	2	2	0	4	2	0	0	2	0	1	0	2	2	0	1	2	2	0	1	4	**70**

Average	71.08%																								

The bold values are to differentiate the original results from the missing results.

The article "A Precise Medical Imaging Approach for Brain MRI Image Classification" was retracted in 2023. Reasons: signs of a paper mill; compromised peer review; unreliable results or conclusions.

**Table 4:** Classification results of kernel principal component analysis (without using the proposed technique) on the brain MRI dataset (unit %).

Diseases	NB	GL	SR	AL	AV	PD	HD	M	CS	MS	CT	HE	MB	MA	MN	CC	AD	LE	CJ	HY	MI	CH	CA	VD	FT
NB	**75**	0	2	1	0	2	2	0	1	1	2	0	4	0	1	2	2	0	1	1	0	2	0	0	1
GL	1	**78**	0	2	2	0	1	1	1	0	2	1	0	1	2	0	0	2	2	0	1	0	1	2	0
SR	0	2	**79**	0	1	1	0	1	2	2	0	0	2	0	0	1	1	0	1	2	0	2	0	1	2
AL	2	0	1	**73**	0	2	2	0	0	1	2	4	0	1	2	0	2	1	0	1	2	0	2	0	2
AV	1	2	0	2	**74**	0	0	2	2	0	2	1	2	0	2	1	0	0	2	2	0	1	2	2	0
PD	0	2	2	0	4	**71**	1	0	1	2	0	0	1	2	0	2	2	2	0	2	1	2	0	2	1
HD	2	0	0	1	1	1	**81**	2	0	0	1	2	0	0	1	0	0	1	2	0	0	1	2	0	2
M	1	2	1	0	0	1	2	**80**	2	0	0	0	1	1	0	2	1	0	0	2	1	0	1	2	0
CS	0	1	0	2	2	0	0	1	**78**	2	2	1	0	0	2	0	0	2	1	0	2	2	0	1	1
MS	2	0	2	0	1	2	2	0	0	**74**	1	2	2	0	0	2	1	0	2	2	0	1	2	0	2
CT	1	2	0	1	2	0	1	2	2	0	**72**	0	1	2	1	0	0	4	0	2	2	0	2	2	1
HE	0	1	2	0	0	1	0	2	0	2	2	**80**	0	0	2	1	1	0	2	0	1	2	0	1	0
MB	2	0	0	4	0	2	1	0	1	0	1	2	**73**	2	0	2	2	1	0	1	2	0	1	1	2
MA	2	1	1	0	2	0	0	2	0	1	1	0	2	**77**	2	0	0	2	1	1	0	2	0	2	1
MN	0	2	0	2	0	2	1	0	2	0	0	1	2	0	**79**	2	1	0	1	2	2	0	1	0	0
CC	2	0	2	0	1	0	2	1	0	2	1	2	0	2	1	**75**	0	2	2	0	0	1	2	0	2
AD	0	1	0	2	0	2	0	1	2	0	0	0	1	1	0	2	**82**	1	0	1	1	0	0	2	1
LE	2	0	1	0	2	0	1	0	1	2	1	1	0	0	2	0	0	**84**	0	0	0	1	2	0	0
CJ	0	2	0	1	0	1	0	2	0	0	0	0	1	2	0	2	2	0	**85**	0	1	0	0	1	0
HY	1	0	2	0	2	2	0	1	1	2	1	0	0	1	2	0	0	2	2	**75**	2	0	1	2	1
MI	2	2	0	1	0	2	1	2	1	0	2	2	2	0	1	1	2	0	1	2	**71**	2	0	1	2
CH	0	1	4	0	2	0	2	1	0	2	1	0	1	2	0	2	0	2	0	4	4	**69**	2	0	1
CA	2	0	1	1	0	2	0	2	6	0	0	2	1	0	4	0	2	1	2	0	1	2	**67**	2	2
VD	2	2	0	0	4	0	2	1	0	1	2	0	0	6	0	2	1	0	1	2	1	0	6	**65**	2
FT	0	1	2	2	0	1	2	0	1	2	0	4	2	0	1	0	2	6	0	2	0	2	0	4	**66**

Average	75.32%																								

The bold values are to differentiate the original results from the missing results.

The article "A Precise Medical Imaging Approach for Brain MRI Image Classification" was retracted in 2023. Reasons: signs of a paper mill; compromised peer review; unreliable results or conclusions.

**Table 5:** Classification results of latent semantic analysis (without using the proposed technique) on the brain MRI dataset (unit %).

Diseases	NB	GL	SR	AL	AV	PD	HD	M	CS	MS	CT	HE	MB	MA	MN	CC	AD	LE	CJ	HY	MI	CH	CA	VD	FT
NB	**78**	1	2	0	2	0	2	0	1	1	2	0	2	0	2	0	2	1	0	1	0	1	0	2	0
GL	2	**80**	0	2	0	1	0	2	2	0	0	1	0	2	0	1	0	0	2	0	2	0	2	0	1
SR	0	2	**82**	0	1	0	1	0	0	2	2	0	1	0	2	0	0	2	0	2	0	1	0	2	0
AL	1	0	2	**86**	0	2	0	0	1	0	0	2	0	1	0	0	2	0	0	0	1	0	1	0	1
AV	2	1	0	2	**74**	0	2	2	0	2	1	0	2	0	2	1	0	1	2	0	0	2	0	2	2
PD	0	2	2	0	2	**72**	0	1	1	0	1	2	1	2	0	0	2	4	0	1	2	0	2	2	1
HD	1	0	3	1	0	2	**77**	0	2	2	0	1	0	1	1	2	0	0	1	2	0	1	2	1	0
M	2	1	0	0	1	0	2	**80**	2	0	1	0	2	0	2	0	1	2	0	0	1	0	1	0	2
CS	0	0	1	2	0	1	0	2	**85**	1	0	2	0	1	0	1	0	0	2	0	0	2	0	0	0
MS	2	1	0	0	1	0	2	0	1	**81**	2	0	1	0	2	0	2	0	0	1	2	0	1	0	1
CT	0	2	2	0	0	2	0	1	0	2	**79**	1	0	2	0	2	0	1	2	0	0	1	0	2	1
HE	1	2	0	2	2	0	1	0	2	0	1	**76**	2	0	1	0	2	2	0	2	1	0	1	0	2
MB	2	0	1	0	2	1	0	2	0	1	2	0	**73**	2	0	1	0	1	2	0	4	2	0	2	2
MA	0	1	0	2	0	2	1	0	1	2	0	2	0	**80**	2	0	2	1	0	1	0	1	1	1	0
MN	2	0	2	0	1	0	0	2	0	1	1	0	2	0	**79**	2	0	0	2	1	2	0	2	0	1
CC	1	2	0	1	0	2	2	0	2	2	0	1	1	2	0	**69**	4	2	0	3	1	2	0	2	1
AD	0	0	1	0	2	0	0	1	0	0	2	0	0	0	2	0	**88**	0	1	1	0	0	1	1	0
LE	1	2	0	1	0	2	1	0	2	1	0	2	2	0	0	1	1	**76**	0	2	2	0	2	0	2
CJ	2	0	2	0	4	2	0	2	1	0	1	2	0	6	2	0	1	2	**68**	0	1	1	0	2	1
HY	1	1	0	2	2	0	2	1	0	2	0	1	1	0	1	2	0	2	4	**71**	2	0	2	1	2
MI	0	2	2	0	1	1	1	0	2	0	2	1	0	2	2	0	2	0	1	2	**75**	2	0	1	1
CH	2	0	1	1	0	2	0	2	0	1	1	0	2	0	0	1	1	4	0	1	2	**72**	6	1	0
CA	1	1	0	1	2	0	2	1	2	0	0	2	1	2	0	2	0	1	2	0	1	2	**75**	0	2
VD	0	2	2	0	1	1	1	0	1	2	2	0	0	1	2	0	2	0	1	2	0	1	2	**76**	1
FT	2	0	1	2	0	0	1	2	0	0	1	1	1	0	0	1	0	2	1	0	2	0	1	2	**80**

Average	77.28%																								

The bold values are to differentiate the original results from the missing results.

**Table 6:** Classification results of partial least squares (without using the proposed technique) on the brain MRI dataset (unit %).

Diseases	NB	GL	SR	AL	AV	PD	HD	M	CS	MS	CT	HE	MB	MA	MN	CC	AD	LE	CJ	HY	MI	CH	CA	VD	FT
NB	**61**	2	2	0	4	2	0	1	6	2	0	2	2	1	0	1	5	2	0	3	1	0	2	1	0
GL	2	**67**	0	2	2	0	2	2	0	1	2	0	1	6	2	0	1	1	2	0	2	2	0	2	1
SR	1	1	**71**	2	0	2	0	1	1	0	4	2	0	1	2	2	0	2	1	2	0	1	2	0	2
AL	0	2	2	**68**	1	1	2	0	2	2	0	2	4	0	1	2	2	0	1	2	2	0	1	2	1
AV	2	0	4	1	**73**	2	1	2	0	1	2	0	1	2	0	1	1	2	0	0	1	2	0	2	0
PD	1	1	0	2	2	**75**	0	1	2	0	1	1	0	2	2	0	0	1	2	2	0	1	2	0	2
HD	0	2	2	0	1	2	**78**	2	1	2	0	0	2	0	0	1	2	0	1	0	1	0	2	1	0
M	2	0	1	2	0	1	2	**69**	1	1	2	4	0	1	2	2	0	2	0	2	2	1	0	2	1
CS	1	4	0	2	2	2	0	2	**67**	2	1	0	2	4	0	1	2	0	1	0	1	2	2	0	2
MS	0	2	2	0	0	1	2	1	1	**71**	2	2	0	0	2	2	1	2	0	2	2	0	4	1	0
CT	2	0	1	2	1	0	1	0	2	2	**70**	1	4	2	0	2	2	1	1	0	1	2	0	2	1
HE	1	2	1	0	2	2	0	2	0	1	1	**74**	0	1	1	0	1	2	2	2	0	1	2	0	2
MB	1	2	0	1	0	1	2	0	1	0	2	2	**77**	0	2	2	0	0	1	2	2	0	1	1	0
MA	0	0	2	2	1	0	0	1	0	2	0	1	2	**79**	0	1	2	2	0	0	1	2	0	0	2
MN	2	1	0	0	2	2	1	0	1	0	1	0	0	2	**81**	0	0	0	2	2	0	0	1	2	0
CC	1	0	2	1	1	1	2	2	0	2	0	5	2	0	2	**67**	2	1	0	2	2	1	0	2	2
AD	2	2	0	2	0	2	1	1	4	0	2	1	1	4	2	2	**66**	0	2	0	0	2	2	1	1
LE	0	2	2	0	2	0	0	4	1	2	0	2	1	1	0	2	4	**69**	0	1	2	1	0	2	2
CJ	2	0	1	2	1	0	1	2	0	1	2	0	2	1	2	0	2	4	**71**	2	0	2	1	0	1
HY	1	2	0	1	2	2	1	0	2	0	0	1	2	0	2	2	0	1	2	**73**	2	0	2	1	1
MI	0	1	2	0	0	1	2	2	0	2	2	2	0	2	0	1	1	2	1	0	**75**	2	0	2	0
CH	2	2	0	2	1	0	0	1	2	0	0	1	2	0	1	0	1	1	0	2	2	**77**	1	0	2
CA	1	1	2	0	1	2	2	0	0	1	2	0	0	1	2	1	0	0	1	1	0	2	**78**	2	0
VD	1	0	0	2	0	0	1	2	2	0	0	2	1	2	0	0	2	1	0	0	1	1	0	**81**	1
FT	0	2	2	0	2	1	0	2	0	2	1	2	0	0	4	2	0	0	2	1	2	0	2	1	**72**

Average	72.40%																								

The bold values are to differentiate the original results from the missing results.

The article "A Precise Medical Imaging Approach for Brain MRI Image Classification" was retracted in 2023. Reasons: signs of a paper mill; compromised peer review; unreliable results or conclusions.

**Table 7:** Classification results of multifactor dimensionality reduction (without using the proposed technique) on the brain MRI dataset (unit %).

Diseases	NB	GL	SR	AL	AV	PD	HD	M	CS	MS	CT	HE	MB	MA	MN	CC	AD	LE	CJ	HY	MI	CH	CA	VD	FT
NB	**70**	2	1	0	1	2	2	0	2	0	1	1	0	4	2	0	1	2	0	2	2	0	2	1	2
GL	2	**67**	2	2	0	0	1	4	1	2	0	2	2	0	1	2	0	2	6	0	1	2	0	1	0
SR	1	0	**69**	1	4	2	0	1	0	2	2	0	1	2	0	2	4	0	2	1	0	2	2	0	2
AL	0	2	2	**72**	1	1	2	0	2	0	1	2	0	1	2	0	2	1	0	2	2	0	2	2	1
AV	2	1	0	2	**74**	0	1	2	0	1	0	2	2	0	2	1	0	2	2	0	0	1	1	2	2
PD	2	0	2	0	1	**66**	0	2	4	0	2	0	1	2	0	6	2	0	1	2	2	1	0	2	2
HD	1	2	0	6	1	2	**62**	1	2	2	0	4	0	1	2	0	2	4	0	2	1	2	2	0	1
M	0	2	4	2	0	2	2	**63**	0	1	2	0	2	4	1	2	0	2	2	0	4	2	1	2	0
CS	2	0	2	2	2	0	4	2	**65**	0	1	2	2	0	2	1	2	0	2	4	0	0	2	1	2
MS	1	2	0	0	1	2	0	1	2	**72**	2	0	1	2	2	0	2	2	0	0	1	1	0	2	4
CT	0	1	2	1	0	0	2	0	2	2	**74**	2	1	0	1	2	0	1	1	2	0	2	2	0	2
HE	2	0	1	2	4	0	1	2	0	1	4	**63**	2	2	0	1	2	2	0	1	6	1	0	1	2
MB	2	2	0	1	2	6	0	1	2	0	2	2	**61**	3	2	0	1	2	4	0	2	2	1	0	2
MA	1	2	2	0	2	1	2	0	1	5	0	1	2	**66**	0	2	2	0	1	2	0	4	2	2	0
MN	2	1	0	2	0	2	0	2	4	0	2	2	0	1	**68**	0	2	2	0	2	4	1	0	2	1
CC	0	2	1	0	4	0	1	2	0	2	0	2	2	0	4	**71**	1	0	2	1	1	0	2	0	2
AD	2	0	2	1	0	1	0	1	1	0	1	0	2	2	0	2	**77**	2	0	2	1	2	0	1	0
LE	2	1	0	4	2	0	2	0	2	1	2	1	0	2	2	0	2	**64**	2	2	0	1	2	4	2
CJ	0	2	2	0	1	4	0	2	1	0	1	2	2	0	1	2	0	1	**72**	0	2	4	0	0	1
HY	1	0	2	1	0	2	3	0	2	2	0	0	1	2	0	2	2	0	2	**69**	4	0	2	1	2
MI	2	2	0	2	2	0	1	2	2	0	2	1	2	0	2	0	1	2	0	2	**70**	2	0	2	1
CH	2	2	1	0	1	6	0	2	0	1	1	6	0	2	2	1	0	3	1	0	2	**62**	1	2	2
CA	0	1	2	2	0	2	2	0	1	0	2	2	1	2	0	2	2	0	2	1	0	4	**70**	0	2
VD	1	0	2	1	2	0	1	2	0	2	1	0	2	0	1	2	0	1	0	2	2	0	2	**76**	0
FT	0	2	0	2	1	1	0	1	2	0	0	2	0	2	0	0	1	2	0	0	2	2	0	2	**78**

Average	68.84%																								

The bold values are to differentiate the original results from the missing results.

The article "A Precise Medical Imaging Approach for Brain MRI Image Classification" was retracted in 2023. Reasons: signs of a paper mill; compromised peer review; unreliable results or conclusions.

**Table 8:** Classification results of nonlinear dimensionality reduction (without using the proposed technique) on the brain MRI dataset (unit %).

Diseases	NB	GL	SR	AL	AV	PD	HD	M	CS	MS	CT	HE	MB	MA	MN	CC	AD	LE	CJ	HY	MI	CH	CA	VD	FT
NB	**80**	0	2	0	1	1	2	0	2	2	0	1	2	1	0	0	1	0	2	0	0	1	0	2	0
GL	1	**84**	0	2	0	0	1	1	0	0	2	0	0	0	2	1	0	0	0	1	2	0	1	0	2
SR	2	1	**73**	0	2	2	0	2	1	1	0	2	3	2	0	0	2	1	2	0	1	2	0	1	0
AL	0	2	2	**76**	0	1	2	0	2	2	1	0	0	1	2	2	0	2	0	2	0	0	2	0	1
AV	1	0	1	2	**79**	0	1	2	0	0	2	1	2	0	0	1	1	0	2	0	2	1	0	2	0
PD	0	1	0	0	2	**85**	0	0	1	2	0	0	0	2	1	0	0	2	0	1	0	0	1	0	2
HD	2	0	2	0	0	0	**89**	1	0	0	1	0	2	0	0	0	1	0	0	0	0	1	0	1	0
M	1	2	0	1	2	2	0	**77**	2	2	0	1	0	0	2	2	0	0	2	1	2	0	1	0	0
CS	0	1	2	2	0	1	2	2	**74**	0	2	0	2	1	1	0	1	2	1	0	0	2	0	2	2
MS	2	0	1	1	2	0	0	1	2	**78**	0	1	0	2	0	2	2	0	0	2	1	0	2	0	1
CT	0	2	0	0	1	2	2	0	0	2	**80**	2	2	0	1	0	0	1	2	0	0	2	0	1	0
HE	1	0	2	2	0	0	0	1	1	0	2	**82**	0	2	0	1	2	0	0	1	2	0	0	0	1
MB	0	1	0	0	1	2	2	0	0	1	0	1	**84**	0	2	0	0	2	1	0	0	1	2	0	0
MA	2	0	2	0	0	0	0	1	0	0	1	0	0	**88**	0	2	1	0	0	0	1	0	0	2	0
MN	0	1	0	1	2	0	0	0	2	0	0	0	1	0	**89**	0	0	0	2	0	0	0	0	0	2
CC	1	0	1	2	0	1	2	2	0	1	2	0	0	1	0	**82**	0	1	0	1	0	2	1	0	0
AD	0	2	1	0	1	0	0	1	1	0	0	2	2	0	2	1	**80**	0	2	0	2	0	0	2	1
LE	2	0	0	2	0	2	2	0	0	2	1	1	0	2	1	0	2	**75**	2	1	0	1	2	0	2
CJ	2	1	2	0	1	2	0	2	2	0	0	2	1	1	0	2	1	2	**73**	0	2	1	0	1	2
HY	1	2	0	1	4	0	1	2	0	1	2	0	3	2	1	0	2	1	1	**70**	1	0	2	2	1
MI	2	0	2	2	0	1	2	0	1	2	0	1	2	0	2	2	0	1	4	2	**69**	2	1	2	0
CH	0	1	1	2	2	1	0	2	2	0	1	2	0	1	0	1	2	2	0	2	0	**74**	2	0	2
CA	2	2	0	1	2	0	2	1	0	2	2	0	2	2	1	0	1	0	2	1	2	0	**73**	2	0
VD	1	2	2	0	0	2	1	2	2	0	0	1	1	0	2	4	0	2	1	0	1	2	1	**71**	2
FT	2	0	1	2	2	1	0	0	1	2	2	0	0	1	0	1	2	1	0	2	0	1	0	1	**78**

Average	78.52%																								

The bold values are to differentiate the original results from the missing results.

**Table 9:** Classification results of multilinear principal component analysis (without using the proposed technique) on the brain MRI dataset (unit %).

Diseases	NB	GL	SR	AL	AV	PD	HD	M	CS	MS	CT	HE	MB	MA	MN	CC	AD	LE	CJ	HY	MI	CH	CA	VD	FT
NB	**82**	1	0	2	0	1	0	2	1	1	0	1	0	1	0	2	0	1	0	2	0	1	0	2	0
GL	2	**77**	1	0	2	0	2	1	0	2	1	0	2	0	1	0	2	0	2	0	1	0	2	0	2
SR	0	1	**89**	1	0	2	0	0	2	0	0	1	0	2	0	1	0	0	0	1	0	0	0	0	0
AL	1	0	0	**90**	1	0	1	0	0	0	2	0	0	0	0	0	0	2	0	0	0	2	0	1	0
AV	0	2	2	0	**78**	1	0	2	1	1	0	2	1	1	2	0	1	0	2	0	2	0	1	0	1
PD	2	0	0	1	0	**82**	2	0	0	2	1	0	2	0	1	2	0	1	0	1	0	1	0	2	0
HD	0	1	0	0	2	0	**86**	1	2	0	0	1	0	1	0	0	2	0	1	0	1	0	0	0	2
M	1	0	2	0	0	1	0	**84**	0	1	2	0	1	0	2	0	0	1	0	2	0	2	0	1	0
CS	0	2	0	1	2	0	2	0	**79**	0	1	2	0	2	0	1	2	0	2	0	2	0	1	0	1
MS	0	0	1	0	0	2	0	1	0	**88**	0	0	1	0	2	0	0	1	0	1	0	1	0	2	0
CT	2	1	0	2	1	0	1	0	2	2	**74**	1	0	1	1	2	2	0	1	0	1	2	2	0	2
HE	0	0	2	0	0	1	0	2	0	0	2	**89**	1	0	0	0	0	1	0	1	0	0	0	1	0
MB	0	1	0	0	2	0	0	0	0	1	0	0	**91**	0	2	0	0	0	2	0	0	0	1	0	0
MA	2	0	1	2	0	2	1	0	1	0	1	2	0	**77**	0	1	2	2	0	0	1	2	0	2	1
MN	0	2	0	1	1	0	2	2	0	2	0	0	2	0	**81**	0	0	0	1	2	0	0	2	0	2
CC	1	0	2	0	2	1	0	0	2	0	2	1	0	2	0	**83**	1	0	0	0	2	0	0	1	0
AD	0	1	0	1	0	0	2	1	0	1	0	2	1	0	2	2	**82**	1	0	1	0	2	0	0	1
LE	2	1	1	0	1	2	0	2	1	0	1	0	2	2	0	1	1	**74**	2	0	2	0	2	1	2
CJ	1	0	2	2	0	1	1	0	2	2	0	1	0	1	2	0	2	2	**75**	2	0	1	1	0	2
HY	0	2	0	0	2	0	2	1	0	1	1	0	2	0	0	1	0	0	0	**85**	1	0	0	2	0
MI	2	0	1	1	0	2	0	0	2	0	0	2	0	2	1	0	0	1	1	0	**83**	2	0	0	0
CH	0	1	0	2	1	0	0	0	0	1	0	0	0	0	0	0	1	0	0	2	0	**89**	1	0	2
CA	1	0	2	0	0	0	2	0	0	0	2	0	1	0	0	2	0	0	0	0	1	0	**87**	2	0
VD	2	2	0	1	2	1	0	1	2	2	0	2	0	1	2	0	2	0	1	1	0	2	0	**75**	1
FT	0	1	2	0	1	2	2	0	0	1	1	0	2	1	0	1	1	2	0	2	2	0	2	1	**76**

Average	82.24%																								

The bold values are to differentiate the original results from the missing results.

The article "A Precise Medical Imaging Approach for Brain MRI Image Classification" was retracted in 2023. Reasons: signs of a paper mill; compromised peer review; unreliable results or conclusions.

**Table 10:** Classification results of multilinear subspace learning (without using the proposed technique) on the brain MRI dataset (unit %).

Diseases	NB	GL	SR	AL	AV	PD	HD	M	CS	MS	CT	HE	MB	MA	MN	CC	AD	LE	CJ	HY	MI	CH	CA	VD	FT
NB	**66**	2	1	0	2	2	2	0	1	4	2	0	1	2	0	2	2	1	0	2	3	0	1	2	2
GL	2	**71**	2	2	0	0	1	2	0	1	1	2	0	1	2	0	2	2	2	0	1	2	0	2	2
SR	0	1	**78**	1	2	1	0	1	2	0	2	1	2	0	2	1	0	0	2	1	0	2	1	0	0
AL	1	2	0	**72**	1	2	2	0	1	2	0	0	1	2	0	0	1	4	0	2	2	0	2	2	1
AV	2	0	2	1	**63**	3	1	2	0	1	2	2	0	1	6	2	0	2	1	0	2	1	0	2	4
PD	3	1	2	0	4	**66**	0	2	2	0	1	2	1	0	1	2	2	0	2	1	0	4	2	0	2
HD	0	2	0	2	1	2	**74**	0	2	2	0	0	2	2	2	0	1	1	0	2	1	0	2	1	1
M	1	1	1	2	0	1	2	**72**	0	1	2	1	0	2	0	4	0	2	2	0	2	1	0	2	1
CS	2	0	2	0	2	1	1	0	**78**	0	1	2	2	0	1	0	2	0	0	1	2	0	2	1	0
MS	0	2	0	1	0	2	2	2	1	**79**	0	0	1	1	0	2	0	1	2	0	0	2	0	0	2
CT	2	1	2	0	1	0	0	2	0	2	**77**	2	0	2	1	0	1	0	0	2	2	0	1	2	0
HE	0	1	0	2	0	1	1	0	2	0	2	**80**	2	0	0	2	0	2	1	0	0	1	2	0	1
MB	2	2	1	0	2	0	1	1	0	2	1	1	**71**	4	2	0	2	0	0	2	2	1	0	1	2
MA	1	0	2	1	0	2	2	2	1	0	2	2	1	**72**	0	1	2	2	2	0	0	2	2	0	1
MN	2	2	0	2	1	1	0	1	2	4	0	1	2	2	**63**	2	0	4	0	1	3	0	4	2	1
CC	2	1	2	0	2	0	2	0	2	2	1	0	0	2	1	**74**	2	0	2	0	2	2	0	1	0
AD	1	2	0	1	0	2	1	2	0	0	2	1	1	0	2	1	**76**	2	0	2	0	1	2	0	1
LE	0	1	2	0	1	0	0	0	1	2	0	2	0	1	0	0	2	**84**	1	0	2	0	0	1	0
CJ	1	0	0	2	0	0	1	0	0	0	1	0	2	0	1	2	0	0	**88**	1	0	0	1	0	0
HY	0	0	1	0	2	1	0	1	2	0	0	0	0	2	0	0	0	1	0	**86**	0	2	0	0	2
MI	2	2	0	1	0	0	4	2	0	2	0	2	1	0	2	1	2	0	2	0	**73**	0	2	2	0
CH	1	0	2	2	1	2	0	0	1	1	2	0	2	1	0	2	0	2	0	2	2	**75**	0	1	1
CA	0	1	1	0	2	0	1	2	2	0	0	1	0	2	1	0	1	2	1	0	2	2	**77**	0	2
VD	2	0	0	2	0	1	0	0	0	1	2	0	1	0	0	2	0	0	1	2	0	0	2	**84**	0
FT	0	2	1	0	0	0	2	0	1	0	0	0	0	1	0	0	0	1	0	0	0	2	0	0	**90**

Average	75.56%																								

The article "A Precise Medical Imaging Approach for Brain MRI Image Classification" was retracted in 2023. Reasons: signs of a paper mill; compromised peer review; unreliable results or conclusions.

**Table 11:** Classification results of semidefinite embedding (without using the proposed technique) on the brain MRI dataset (unit %).

Diseases	NB	GL	SR	AL	AV	PD	HD	M	CS	MS	CT	HE	MB	MA	MN	CC	AD	LE	CJ	HY	MI	CH	CA	VD	FT
NB	**59**	2	0	2	1	2	0	2	6	4	3	0	2	1	4	0	2	1	0	2	2	0	1	2	2
GL	2	**63**	4	0	2	1	2	0	2	1	2	2	0	2	1	2	0	2	4	0	1	2	0	4	1
SR	1	2	**71**	2	0	2	1	2	0	2	0	2	1	2	0	1	2	0	1	2	0	2	2	0	2
AL	0	1	2	**73**	1	0	1	2	2	0	1	1	2	0	2	0	2	1	0	2	2	0	4	1	0
AV	2	0	1	4	**63**	2	0	5	2	2	4	0	0	1	2	2	0	2	1	0	3	1	0	2	1
PD	0	2	2	0	1	**74**	2	2	0	1	0	2	2	2	0	2	1	0	2	1	0	2	1	0	1
HD	2	1	0	2	2	1	**66**	0	1	2	2	0	1	0	2	0	2	4	0	2	1	6	1	2	0
M	1	0	2	0	0	2	1	**78**	2	0	1	2	0	1	0	1	0	2	2	0	2	0	0	1	2
CS	0	2	0	1	2	0	0	2	**80**	2	0	0	2	0	1	0	2	0	0	1	0	1	2	0	2
MS	2	0	1	2	0	1	2	0	2	**77**	2	1	0	2	2	1	0	1	2	0	1	0	0	1	0
CT	2	1	2	0	1	2	0	1	2	2	**64**	2	4	0	1	2	6	0	0	2	0	2	1	2	1
HE	1	2	0	2	2	0	1	2	0	1	2	**67**	2	4	0	2	1	2	2	0	1	2	2	0	2
MB	0	2	1	2	0	2	2	0	1	2	1	2	**71**	2	1	0	2	1	0	1	3	0	2	1	1
MA	2	0	2	0	1	2	0	2	2	0	2	1	2	**65**	2	4	0	2	1	4	0	2	0	2	2
MN	1	2	0	1	2	0	1	1	0	2	0	2	2	2	**73**	0	1	0	2	1	2	0	1	2	2
CC	0	2	2	1	0	1	2	0	2	0	1	1	0	2	2	**72**	2	1	0	2	1	2	0	4	0
AD	2	0	1	2	2	2	0	1	0	2	2	0	1	0	2	2	**75**	0	2	0	0	1	2	0	1
LE	2	1	2	0	1	0	2	2	1	0	0	2	2	4	0	2	1	**66**	4	1	2	0	1	2	2
CJ	0	2	0	2	2	1	0	1	2	2	4	0	1	2	1	0	2	2	**69**	2	0	3	0	1	1
HY	1	2	1	0	0	2	2	0	1	2	0	2	0	1	2	2	0	1	2	**72**	2	1	2	0	2
MI	2	0	2	1	1	0	2	2	0	1	2	1	2	0	1	1	4	0	1	2	**69**	2	0	2	2
CH	2	1	0	2	2	1	0	1	2	0	1	2	1	2	0	0	2	2	0	0	1	**74**	2	2	0
CA	0	2	1	0	1	0	1	0	1	2	0	0	0	1	2	2	0	0	2	1	0	1	**81**	0	2
VD	1	0	2	2	0	2	0	2	0	1	2	4	2	0	1	3	2	4	1	0	2	2	2	**64**	1
FT	2	1	0	1	3	0	4	1	2	0	2	1	0	2	2	0	1	2	0	2	4	0	1	6	**63**

Average	69.96%																								

**Table 12:** Comparison of the proposed technique with state-of-the-art methods against MRI images.

Systems	Accuracies (%)	Standard deviation
[45]	75.8	±3.8
[46]	82.5	±4.4
[47]	87.6	±2.8
[48]	70.1	±5.7
[49]	89.9	±3.0
[50]	77.7	±4.9
[51]	90.4	±1.1
[52]	81.7	±2.6
[53]	74.2	±3.1
[54]	91.3	±0.9
Proposed technique	96.4	±3.6

The article "A Precise Medical Imaging Approach for Brain MRI Image Classification" was retracted in 2023. Reasons: signs of a paper mill; compromised peer review; unreliable results or conclusions.

## Data Availability

The data used for this study and simulation will be provided on demand.

## References

[1] UN News (2022). Global perspective Human stories. https://news.un.org/en/story/2007/02/210312.

[2] Siddiqui M. F., Reza A. W., Kanesan J. (2015). An automated and intelligent medical decision support system for brain MRI scans classification. *PLoS One*.

[3] Maji P., Chanda B., Kundu M. K., Dasgupta S. Deformation correction in brain MRI using mutual information and genetic algorithm.

[4] Zhang Y. D., Wu L., Wang S. (2011). Magnetic resonance brain image classification by an improved artificial bee colony algorithm. *Progress In Electromagnetics Research*.

[5] Mwangi B., Ebmeier K. P., Matthews K., Douglas Steele J. (2012). Multi-centre diagnostic classification of individual structural neuroimaging scans from patients with major depressive disorder. *Brain*.

[6] Klöppel S., Stonnington C. M., Barnes J. (2008). Accuracy of dementia diagnosis—a direct comparison between radiologists and a computerized method. *Brain*.

[7] Faisal A., Parveen S., Badsha S., Sarwar H., Reza A. W. (2013). Computer assisted diagnostic system in tumor radiography. *Journal of Medical Systems*.

[8] Shaji S., Ganapathy N., Swaminathan R. (2021). Classification of alzheimer condition using MR brain images and inception-residual network model. *Current Directions in Biomedical Engineering*.

[9] Khagi B., Kwon G. R. (2021). 3D CNN based Alzheimer’s diseases classification using segmented Grey matter extracted from whole-brain MRI. *JOIV: International Journal on Informatics Visualization*.

[10] Tinauer C., Heber S., Pirpamer L. (2021). *Explainable Brain Disease Classification and Relevance-Guided Deep Learning*.

[11] Zhou C., Ding C., Wang X., Lu Z., Tao D. (2020). One-pass multi-task networks with cross-task guided attention for brain tumor segmentation. *IEEE Transactions on Image Processing*.

[12] Yang Y., Yan L. F., Zhang X. (2018). Glioma grading on conventional MR images: a deep learning study with transfer learning. *Frontiers in Neuroscience*.

[13] Thayumanavan M., Ramasamy A. (2021). An efficient approach for brain tumor detection and segmentation in MR brain images using random forest classifier. *Concurrent Engineering*.

[14] Sevli O. (2021). Performance comparison of different pre-trained deep learning models in classifying brain MRI images. *Acta Infologica*.

[15] Gull S., Akbar S., Khan H. U. (2021). Automated Detection of Brain Tumor through Magnetic Resonance Images Using Convolutional Neural Network. *BioMed Research International*.

[16] Med.Harvard (2022). Harvard Medical School. http://med.harvard.edu/AANLIB/.

The article "A Precise Medical Imaging Approach for Brain MRI Image Classification" was retracted in 2023. Reasons: signs of a paper mill; compromised peer review; unreliable results or conclusions.

[17] Oasis-Brains (2022). Open access series of imaging studies. http://www.oasis-brains.org/.

[18] Hamzenejad A., Ghoushchi S. J., Baradaran V. (2021). Clustering of Brain Tumor Based on Analysis of MRI Images Using Robust Principal Component Analysis (ROBPCA) Algorithm. *BioMed Research International*.

[19] Georgieva P., De la Torre F. Robust principal component analysis for brain imaging.

[20] Palki G., Patil A., Kumar S., Perur S. D., Kumar S. (2017). A novel MRI brain images classifier using PCA and SVM. *International Journal of Engineering Research and Technology*.

[21] Topannavar P. S. (2021). Rotational wavelet filters for analysis of brain MRI in detection of Alzheimer’s disease. *Turkish Journal of Computer and Mathematics Education (TURCOMAT)*.

[22] Naser W. A. K., Kadim E. A., Abbas S. H. (2021). SVM Kernels comparison for brain tumor diagnosis using MRI. *Global Journal of Engineering and Technology Advances*.

[23] Bauer S., Nolte L. P., Reyes M. Fully automatic segmentation of brain tumor images using support vector machine classification in combination with hierarchical conditional random field regularization.

[24] Abd El Kader I., Xu G., Shuai Z. (2021). Brain tumor detection and classification on MR images by a deep wavelet auto-encoder model. *Diagnostics*.

[25] Jha D., Kim J. I., Kwon G. R. (2017). Diagnosis of Alzheimer’s disease using dual-tree complex wavelet transform, PCA, and feed-forward neural network. *Journal of healthcare engineering*.

[26] Lee B., Yamanakkanavar N., Choi J. Y. (2020). Automatic segmentation of brain MRI using a novel patch-wise U-net deep architecture. *PLoS One*.

[27] Yamanakkanavar N., Lee B. (2020). Using a patch-wise m-net convolutional neural network for tissue segmentation in brain mri images. *IEEE Access*.

[28] Adiga S., Sivaswamy J. (2019). Fpd-m-net: fingerprint image denoising and inpainting using m-net based convolutional neural networks. *Inpainting and Denoising Challenges*.

[29] Gu X., Shen Z., Xue J., Fan Y., Ni T. (2021). Brain tumor MR image classification using convolutional dictionary learning with local constraint. *Frontiers in Neuroscience*.

[30] Kenyhercz M. W., Passalacqua N. V. (2016). Missing data imputation methods and their performance with biodistance analyses. *Biological Distance Analysis*.

[31] Irmak E. (2021). Multi-classification of brain tumor MRI images using deep convolutional neural network with fully optimized framework. *Iranian Journal of Science and Technology, Transactions of Electrical Engineering*.

[32] Zhang Y., Dong Z., Wu L., Wang S. (2011). A hybrid method for MRI brain image classification. *Expert Systems with Applications*.

The article "A Precise Medical Imaging Approach for Brain MRI Image Classification" was retracted in 2023. Reasons: signs of a paper mill; compromised peer review; unreliable results or conclusions.

[33] Naga Srinivasu P., Balas V. E. (2021). Self-Learning Network-based segmentation for real-time brain MR images through HARIS. *PeerJ Computer Science*.

[34] Fayaz M., Torokeldiev N., Turdumamatov S., Qureshi M. S., Qureshi M. B., Gwak J. (2021). An efficient methodology for brain MRI classification based on DWT and convolutional neural network. *Sensors*.

[35] H Alkinani M., A Zanaty E., M Ibrahim S. (2021). Medical image compression based on wavelets with particle swarm optimization. *Computers, Materials & Continua*.

[36] Abdulameer A. T. (2018). An improvement of MRI brain images classification using dragonfly algorithm as trainer of artificial neural network. *Ibn AL-Haitham Journal for Pure and Applied Science*.

[37] Kumar Das T., Kumar Roy P., Uddin M., Srinivasan K., Chang C. Y., Syed-Abdul S. (2021). Early tumor diagnosis in brain MR images via deep convolutional neural network model. *Computers, Materials & Continua*.

[38] Malathi M., Sinthia P. (2018). MRI brain tumour segmentation using hybrid clustering and classification by back propagation algorithm. *Asian Pacific Journal of Cancer Prevention*.

[39] Mehta N., Sethi P. (2018). K-mean clustering in health care using map reduce. *International Journal of Management, Technology And Engineering*.

[40] Shanmugavadivu P., Kavitha M. S. Data imputation of brain MRI features with enhanced multinomial logistic regression for Alzheimer’s disease classification.

[41] Mika S., Ratsch G., Weston J., Scholkopf B., Mullers K.-R. Fisher discriminant analysis with kernels.

[42] Krusienski D. J., Sellers E., McFarland D., Vaughan T., Wolpaw J. (2008). Toward enhanced P300 speller performance. *Journal of Neuroscience Methods*.

[43] Quantifying Health (2022). Understand Forward and Backward Stepwise Regression. https://quantifyinghealth.com/stepwise-selection/.

[44] Weis M., Rumpf T., Gerhards R., Lutz P. (2009). Comparison of different classification algorithms for weed detection from images based on shape parameters. *Bornimer Agrartechn. Ber*.

[45] Saratxaga C. L., Moya I., Picón A. (2021). MRI deep learning-based solution for Alzheimer’s disease prediction. *Journal of Personalized Medicine*.

[46] Mohammed B. A., Rassem T. H., Makbol N. M. (2021). Multi-method analysis of medical records and MRI images for early diagnosis of dementia and Alzheimer’s disease based on deep learning and hybrid methods. *Electronics*.

[47] Islam J., Zhang Y. (2017). An ensemble of deep convolutional neural networks for Alzheimer’s disease detection and classification. https://arxiv.org/abs/1712.01675.

[48] Maqsood M., Nazir F., Khan U. (2019). Transfer learning assisted classification and detection of Alzheimer’s disease stages using 3D MRI scans. *Sensors*.

The article "A Precise Medical Imaging Approach for Brain MRI Image Classification" was retracted in 2023. Reasons: signs of a paper mill; compromised peer review; unreliable results or conclusions.

[49] Liu J., Li M., Luo Y., Yang S., Li W., Bi Y. (2021). Alzheimer’s disease detection using depthwise separable convolutional neural networks. *Computer Methods and Programs in Biomedicine*.

[50] Bansal D., Khanna K., Chhikara R., Dua R. K., Malhotra R. (2020). Classification of magnetic resonance images using bag of features for detecting dementia. *Procedia Computer Science*.

[51] Leong L. K., Abdullah A. A. (2019). Prediction of Alzheimer’s disease (AD) using machine learning techniques with b algorithm as feature selection method. *Journal of Physics: Conference Series*.

[52] Jain M., Rai C. S., Jain J. (2021). A novel method for differential prognosis of brain degenerative diseases using radiomics-based textural analysis and ensemble learning classifiers. *Computational and Mathematical Methods in Medicine*.

[53] Folego G., Weiler M., Casseb R. F., Pires R., Rocha A. (2020). Alzheimer’s disease detection through whole-brain 3D-CNN MRI. *Frontiers in Bioengineering and Biotechnology*.

[54] Faisal F. U. R., Khatri U., Kwon G.-R. (2021). Diagnosis of Alzheimer’s disease using combined feature selection method. *Journal of Korea Multimedia Society*.

